# Sevoflurane modulates AQPs (1,5) expression and endoplasmic reticulum stress in mice lung with allergic airway inflammation

**DOI:** 10.1042/BSR20193282

**Published:** 2019-11-22

**Authors:** Chang-Ming Lv, Hui-Mei Wu, Ling Wu, Guang-Hong Xu, Zhi-Lai Yang, Qi-Ying Shen

**Affiliations:** 1 Department of Anesthesiology, The First Affiliated Hospital of Anhui Medical University, Hefei 230022, Anhui, China; 2 Department of Geriatric Respiratory and Critical Care, Anhui Geriatric Institute, The First Affiliated Hospital of Anhui Medical University, Hefei, Anhui, China

**Keywords:** Aqps, Asthma, inflammation, Sevoflurane

## Abstract

Sevoflurane was found to show protective roles in mice with asthma, however, the mechanism of which needs further exploring. Aquaporins (AQPs) have been demonstrated to be involved in the pathogenesis of asthma, while endoplasmic reticulum stress has been reported to be related to many inflammatory diseases and involved in protein processing, including AQPs. The present study aimed to determine the role of sevoflurane in AQPs (AQP1,3,4,5) expression in mice with allergic airway inflammation and the probable mechanism. The increased number of inflammatory cells infiltrating the lung tissue, and the elevated levels of tumor necrosis factor-α (TNF-α) and interleukin (IL) 13 (IL-13) were all decreased after sevoflurane treatment (all *P*<0.05). Meanwhile, mRNA levels of AQP1 and AQP5 but not AQP3 and AQP4 were decreased in ovalbumin (OVA)-induced allergic mice lung. Both the decreased mRNA expression and protein levels of AQP1 and AQP5 in allergic lung tissues were reversed by sevoflurane treatment. Furthermore, we established that sevoflurane inhibited the OVA-induced protein increase in the endoplasmic reticulum (ER) stress markers BiP and C/EBP homologous protein (CHOP). Collectively, these findings suggested that sevoflurane modulated the expression and protein level of AOPs (AQP1, AQP5) as well as inhibited ER stress response in OVA-induced allergic airway inflammation of mice.

## Introduction

Asthma is a heterogeneous disorder characterized by variable degrees of inflammation, bronchial hyperreactivity, and airway remodeling [1]. These pathological changes are mediated by several inflammatory cells and cytokines involved in the immune response [2,3]. There are many clinical therapeutic targets for controlling acute asthma at present, and sedatives are considered the last choice of treatment for poorly controlled acute status asthmaticus in the critical care unit setting [4]. The treatment of acute asthma should include both bronchodilators and anti-inflammatory agents. Sevoflurane, a volatile anesthetic agent, has been shown to be effective in controlling severe bronchoconstriction which was ineffective to conventional treatment. Besides, sevoflurane was demonstrated to be helpful in alleviating ovalbumin (OVA)-induced allergic airway inflammation and remodeling in mice [5–7]. Even though, more research still needs to explore how sevoflurane exerts its anti-inflammatory role, in order to provide sufficient basis for the clinical application of sevoflurane in controlling acute asthma.

Aquaporins (AQPs) belong to channel protein, which show a wide distribution in different organs and tissues [8–10]. In recent years, AQPs have been suggested as a target for treatment of many pulmonary diseases, such as cancer, inflammation, and others [11–14]. In lung tissues, there are mainly four types of functional AQPs (AQP1,3,4,5) which attract researchers’ attention. AQP1 is mainly located in pulmonary vascular endothelial cells and interstitial cells, and AQP5 is located in the non-ciliated epithelial cells of the small airways and the apical membranes of type 1 and type 2 airway epithelium. Both AQP1 and AQP5 play crucial roles in maintaining osmolality [15]. The major function of AQP1 is to facilitate water transport between capillary vessel and the alveolar, and AQP5 is to facilitate water transport by osmosis and promote gland secretion [11]. Incremental increases in the osmolality of tracheobronchial lavage fluid have been shown to stimulate the release of inflammatory mediators, indicating a link between fluid homeostasis and inflammation [16]. Some researchers have claimed that the gene expressions of AQP1 and AQP5 are altered in various asthma models [17,18]. Therefore, whether sevoflurane has any effect on the protein levels of AQPs in lung arouse our interest.

Moreover, endoplasmic reticulum (ER) is involved in the post-translational processing of newly synthesized membrane proteins and secretory proteins and attenuating ER stress could reverse the decreased protein level of AQPs in some diseases [19,20]. Researches showed that the decreased AQPs protein levels were correlated with ER stress [21]. Excessive ER stress could result in tissue damage and cell injury, and it has been observed in many inflammatory diseases, including asthma [22,23]. Recent studies indicate that ER stress might be a potential target for controlling inflammatory responses [24]. However, the effect of sevoflurane on ER stress response in asthma is still unknown.

The present study was established to determine the effect of sevoflurane on the expression of AQPs in lungs of mice with OVA-induced allergic airway inflammation. Besides, the influence of sevoflurane on ER stress was also investigated.

## Materials and methods

### Animals and experimental protocol

Female C57BL/6 mice (aged 6–7 weeks) were purchased from SLAC and then housed and treated in Laboratory Animal Center of Anhui Medical University. All animal experiments were approved by the Committee on Animal Welfare at Anhui Medical University (the approval number LLSC20160252).

The mice were randomly divided into three groups: Control (saline treatment); OVA (ovalbumin sensitization/challenge); and OVA+SEV (ovalbumin sensitization/challenge plus sevoflurane treatment). The mice in the OVA and OVA+SEV groups were sensitized (day 0) with an intraperitoneal injection of 10 μg OVA (Sigma, St. Louis, MO, U.S.A.) emulsified in 1 mg alum (Sango Biotech, Shanghai, China). The mice were made to inhale 1% OVA aerosol spray for 30 min/day, from days 14 to 21. In the OVA+SEV group, 3% sevoflurane (Maruishi Pharmaceutical, Osaka, Japan) was administered before each OVA treatment. The mice in the control group received intraperitoneal and aerosol treatments with normal saline only. All mice were killed on day 22. The detailed procedure for setting OVA-induced mice model with allergic airway inflammation was the same as we previously reported [5,6].

### Bronchoalveolar lavage

At 24 h after the last inhalational OVA treatment, the right lung was ligated, and the left lung was subjected to bronchoalveolar lavage with 500 µl phosphate-buffered saline (PBS), which was instilled into the trachea three times via a blunt 22-gauge needle. The right lung was removed and stored at −80°C. The bronchoalveolar lavage fluid (BALF) was centrifuged at 700×***g*** for 5 min. Cells in the lavage fluid were counted using a hemocytometer. Cell differentiation was assessed using Wright–Giemsa staining. The cell-free fractions of BALF aliquots were frozen and stored at −80°C until processed.

### Histopathology

The upper lobe of the right lung was fixed with 10% neutral buffered formalin and embedded in paraffin. Ultrathin sections (4 µm) were obtained. The sections were stained with Hematoxylin and Eosin (HE) and examined microscopically. To demonstrate mucus-secreting goblet cells, Periodic acid–Schiff (PAS) staining was also performed in adjacent sections. Quantitative analysis of PAS-positive areas was performed using Image-Pro Plus 6.0 system.

### Cytokine analysis

ELISA kits were used to measure interleukin (IL)-10, IL-13, and tumor necrosis factor-α (TNF-α) levels (Cusabio, Wuhan, China) in BALF, according to the manufacturer’s instructions.

### RNA extraction and quantitative real-time PCR

Gene expression of AQP1,3,4,5 in lung tissues was measured using quantitative real-time PCR (qPCR). TRIzol reagent (Ambion) was used for extracting total RNA from lung tissues according to the manufacturer’s protocol, and reverse transcription was performed at 37°C for 30 min using PrimeScript™ RT Master Mix (Takara). The primers used are listed as follows: AQP1, forward 5′-TGC GTT CTG GCC ACC ACTGAC-3′ and reverse 5′-GAT GTC GTC AGC ATC CAG GTC-3′; AQP3, forward 5′-CTG GAC GCT TTC ACT GTG GGC-3′ and reverse 5′-GAT CTG CTC CTT GTG TTT CAT G-3′; AQP4, forward 5′-CTG GAG CCA GCA TGA ATC CAG-3′ and reverse 5′-TTC TTC TCT TCC CAC GGT CA-3′; AQP5, forward 5′-CTC TGC ATC TTC TCC TCC ACG-3′ and reverse 5′-TCC TCT CTA TGA TCT TCC CAG-3′; GAPDH, forward 5′-ACC ACA GTC CAT GCC ATC AC-3′ and reverse 5′-TCC ACC ACC CTG TTG CTG TA-3′.

### Immunohistochemistry

Paraffin-embedded lung tissues were immunostained to visualize AQP1 and AQP5. The tissue sections were dewaxed in toluene, dehydrated in ethanol, rehydrated in double-distilled water, and finally placed in sodium citrate buffer (pH, 6.0) and microwaved twice at 800 W for 4 min each. Endogenous peroxidase in the tissue was blocked by incubation with 1% H_2_O_2_ in PBS at pH 7.4. After immersing the sections in 0.3% Triton-X 100 for 20 min, we incubated them with 5% normal goat serum for 30 min to block non-specific antibodies. The sections were then incubated with anti-AQP1 antibody, anti-AQP5, anti-BiP antibody and anti-C/EBP homologous protein (CHOP) antibody at 4°C for 24 h and washed thrice with PBS for 5 min each. Next, the sections were incubated with peroxidase-labeled secondary antibody for 1 h and washed with PBS again. Horseradish peroxidase (HRP)-labeled streptavidin was added, and the sections were incubated at 37°C for 30 min. After this, the sections were washed with PBS, and diaminobenzidine was used for coloration, followed by counterstaining with Hematoxylin. Finally, the tissue sections were dehydrated and mounted on slides. Quantitative analysis of positive areas was performed using Image-Pro Plus 6.0 system as described in our previous study [5].

### Western blot analysis

Lung tissues were homogenized in RIPA buffer with the presence of protease inhibitors (Roche, Indianapolis, IN, U.S.A.), and protein concentrations were determined. Samples were loaded on to 10% gels for sodium dodecyl sulfate/polyacrylamide gel electrophoresis and transferred to polyvinylidene fluoride membranes (Millipore, Billerica, MA, U.S.A.) by means of the wet transfer method. The membranes were blocked with 5% nonfat milk, and then incubated overnight at 4°C with anti-AQP1 (Abcam, Massachusetts, U.S.A.), anti-AQP5 (Abcam, Massachusetts, U.S.A.), anti-BiP (Proteintech, Rosemont, U.S.A.) and anti-CHOP (Abcam, Massachusetts, U.S.A.) antibody. Anti-rabbit HRP–conjugated IgG was used to detect the bound antibodies. The binding of the specific antibody was visualized using enhanced chemiluminescence (Thermo Scientific, Tewksbury, MA, U.S.A.).

### Statistical analysis

Results are reported as mean ± standard error of the mean (SEM) for the indicated experiments. Statistical comparisons between groups were made using one-way analysis of variance (ANOVA), and then by the Student–Newman–Keuls test, with SPSS16.0. Differences were considered statistically significant at *P*<0.05.

## Results

### Sevoflurane inhibits OVA-induced lung inflammation

In order to confirm the successful setting of the model, and compared the pathological change in lung, HE staining was used to observe airway inflammation. Histopathological analysis of the lung-tissue sections revealed a remarkable difference between the Control group and the OVA group. The sections in the OVA group (Figure 1B) showed greater inflammatory responses with extensive peribronchial, perivascular, and parenchymal inflammatory cells infiltration, and more damaged epithelial cells than those in the Control group (Figure 1A). However, lung-tissue sections from the OVA+SEV group (Figure 1C) showed less inflammation than those in the sections from the OVA group. The number of infiltrating inflammatory cells was decreased, and the alveolar damage was lessened after sevoflurane treatment. These results were also confirmed by the detection of total and differential cells in the BALF (Figure 2).

**Figure 1:** Sevoflurane inhibited OVA-induced lung inflammation Representative hematoxylin and eosin staining (H&E)-stained lung sections are shown (magnification ×200; scale bar, 50 μm). (**A**) Control group; (**B**) OVA group; (**C**) OVA+SEV group.

**Figure 2:** Sevoflurane decreased inflammatory cells in BALF from sensitized mice Total and differential cell counts in BALF sampled from mice 24 h after the last OVA challenge. (**A**) Total cell count in BALF of each group. (**B**–**E**) Differential cell count in BALF, including eosinophils, lymphocytes, neutrophils, and monocytes. Data are presented as the mean ± SEM of each group (*n*=6 per group) from three separate experiments. **P<0.01 vs. control group; ^#^*P*<0.05, ^##^*P*<0.01 vs. OVA group.

The levels of TNF-α, IL-13, and IL-10 in BALF were determined using ELISA kits. Compared with the Control group, levels of TNF-α and IL-13 increased greatly in the OVA group; after treatment with sevoflurane, the levels of TNF-α and IL-13 reduced substantially in the OVA+SEV group as compared with those in the OVA group (Figure 3A,B). The level of IL-10 in BALF showed no statistically difference between the OVA and Control groups, while significantly increased in OVA+SEV group as compared with that in the OVA group (Figure 3C).

**Figure 3:** Sevoflurane modulated levels of cytokines in BALF from sensitized mice ELISA kits were used to detect the protein level of (**A**) TNF-α, (**B**) IL-13, and (**C**) IL-10 in BALF at 24 h after the last challenge. Data are presented as the mean ± SEM of each group (*n*=6 per group) from three separate experiments. *P<0.05 vs. control group; ^#^*P*<0.05 vs. OVA group.

### Sevoflurane alleviates OVA-induced hypertrophied goblet cells and mucus hypersecretion

Hypertrophied goblet cells combined with increased mucus secretion in airway is one of the characteristics of acute allergic airway inflammation. Lung tissues from the OVA group (Figure 4A,B) showed obvious hypertrophy of the goblet cells and increased mucus secretion compared with those in the Control group (Figure 4A(a)). The intensity of PAS staining in the OVA+SEV group (Figure 4A(c)) was less than that in the OVA group. Quantitative analyses revealed that sevoflurane significantly alleviated OVA-induced mucus hypersecretion in allergic mice (*P*<0.01, Figure 4B).

**Figure 4:** Sevoflurane alleviates OVA-induced mucus hypersecretion (**A**) Positively stained hypertrophied goblet cells (shown at the arrows) and magenta staining within the bronchiolar lumen indicates PAS staining of mucus (magnification ×200; scale bar, 50 μm). (**a**) Control group; (**b**) OVA group; (**c**) OVA+SEV group. Abbreviation: BR, bronchus. (**B**) Intensity of PAS positive area is presented as mean ± SEM of each group (*n*=6 per group) from three separate experiments. **P<0.01 vs. control group; ^##^*P*<0.01 vs. OVA group.

### Sevoflurane increased the mRNA and protein levels of AQP1,5 in the lungs of allergic mice

The expression and protein function of some AQPs are critically related to lung disease and function. Here, we detected the mRNA levels of known AQPs (AQP1,2,3,4) in the lung. The mRNA levels of AQP1 and AQP5 in OVA group were significantly lower compared with those in Control group, which were significantly increased in OVA+SEV group (Figure 5A,D). There were no significant differences in the mRNA levels of AQP3 and AQP4 among the three groups (Figure 5B,C).

**Figure 5:** Sevoflurane increased the down-regulated mRNA levels of AQP1,5 in the lungs of allergic mice (**A**–**D**) The mRNA levels of AQP1,3,4,5 in lung tissues from each group were detected by qPCR. Data are presented as the mean ± SEM of each group (*n*=6 per group) from three separate experiments. *P<0.05, **P<0.01 vs. control group; ^#^*P*<0.05, ^##^*P*<0.01 vs. OVA group.

Immunohistochemical staining revealed that protein level of AQP1 was lower in OVA group (Figure 6A(b),B) than that of Control group (Figure 6A(a),B), while was higher in OVA+SEV group (Figure 6A(c),B) than that in OVA group. These results were confirmed by Western blot analysis (Figure 6C,D). Mice in OVA group exhibited lower AQP5 protein level than mice in Control group and OVA+SEV group. The decreased protein level of AQP5 induced by OVA was also reversed by sevoflurane (Figure 7).

**Figure 6:** Sevoflurane reversed the decreased protein level of AQP1 in the lung tissues of allergic mice (**A**) Representative images of AQP1 protein stained by immunohistochemistry in each group are shown (magnification ×100; scale bar, 100 μm). (**a**) Control group; (**b**) OVA group; (**c**) OVA+SEV group. The tan color indicates AQP1-positive staining. (**B**) The quantitative analysis of AQP1 expression. (**C**) AQP1 protein levels in lung tissues were determined using Western blot analysis. (**D**) The results of densitometric analyses are presented as the relative ratio of AQP1 to tubulin. Data are presented as the mean ± SEM of each group (*n*=6 per group) from three separate experiments. *P<0.05 vs. control group; ^#^*P*<0.05 vs. OVA group.

**Figure 7:** Sevoflurane reversed the decreased protein level of AQP5 in the lung tissues of allergic mice (**A**) Representative images of AQP5 protein stained by immunohistochemistry in each group are shown (magnification ×100; scale bar, 100 μm). (**a**) Control group; (**b**) OVA group; (**c**) OVA+SEV group. The tan color indicates AQP5-positive staining. (**B**) The quantitative analysis of AQP5 expression. (**C**) AQP5 protein levels in lung tissues were determined using Western blot analysis. (**D**) The results of densitometric analyses are presented as the relative ratio of AQP5 to tubulin. Data are presented as the mean ± SEM of each group (*n*=6 per group) from three separate experiments. *P<0.05 vs. control group; ^#^*P*<0.05 vs. OVA group.

### Sevoflurane decreased the protein levels of BiP and CHOP in the lung tissues of allergic mice

ER stress has been indicated to contribute to asthma [25]. GRP78 (BiP) and CHOP are the markers of ER stress and increase in many pathological conditions. In the present study, results from immunohistochemical staining and Western blot analysis revealed that the protein levels of both BiP and CHOP significantly increased in OVA group compared with those in Control group, which was in accordance with others’ reports, and treatment with sevoflurane significantly decreased the protein levels of BiP and CHOP (Figure 8).

**Figure 8:** Sevoflurane decreased the protein levels of BiP and CHOP in the lung tissues of allergic mice (**A**) Representative images of BiP protein stained by immunohistochemistry in each group are shown (magnification ×100; scale bar, 100 μm). (**a**) Control group; (**b**) OVA group; (**c**) OVA+SEV group. The tan color indicates BiP-positive staining. (**B**) The quantitative analysis of BiP expression. (**C**) BiP protein levels in lung tissues were determined using Western blot analysis. (**D**) The results of densitometric analyses are presented as the relative ratio of BiP to tubulin. (**E**) Representative images of CHOP protein stained by immunohistochemistry in each group are shown (magnification ×200; scale bar, 100 μm). (**a**) Control group; (**b**) OVA group; (**c**) OVA+SEV group. The tan color indicates CHOP-positive staining. (**F**) The quantitative analysis of CHOP expression. (**G**) CHOP protein levels in lung tissues were determined using Western blot analysis. (**H**) The results of densitometric analyses are presented as the relative ratio of CHOP to tubulin. **P<0.01, ***P<0.001 vs. control group; ^#^*P*<0.05, ^##^*P*<0.01, ^###^*P*<0.001 vs. OVA group.

## Discussion

In clinical and experimental studies, sevoflurane was proved to potently inhibit airway contractility and provide clinical improvement [26–28]. Our previous studies also showed that sevoflurane alleviated OVA-induced airway inflammation in mice, and inhibited T helper 2 (Th2) responses. In the present study, both the expression and protein levels of AQP1 and AQP5 in the lung tissue were lower in the allergic mice than in the control mice and higher in the sevoflurane-treated mice than in the OVA-group mice. Additionally, the increased protein levels of BiP and CHOP induced by OVA were reversed by sevoflurane. These results from this research confirmed the anti-inflammatory role of sevoflurane again.

A skewed Th2 cytokine response with increases in IL-4, IL-6 and IL-13 levels is a salient feature of allergic inflammation in the airway [29–31]. The recruitment and activation of leukocytes, including lymphocytes, monocytes, eosinophils, and neutrophils, leads to bronchial or lung tissue infiltration [32,33]. The following up-regulated release of some pro-inflammatory cytokines could further exacerbate lung inflammation and damage through many routines. In the current study, we determined that sevoflurane reduced inflammatory cell infiltration in BALF and IL-13 and TNF-α production. Sevoflurane also enhanced the production of IL-10. Given the immunosuppressive and anti-inflammatory effects of IL-10 [34,35], the sevoflurane-mediated increase in IL-10 levels improved the imbalance between pro- and anti-inflammatory cytokines response, as reported in our previous study.

Both AQP1 and AQP5 have been regarded as a potential downstream target of inflammatory responses, and its abundance is altered by airway inflammation [36,37]. AQP5 is known to be mostly correlated with abnormal gland secretion in airway. Recent studies have supported the notion that the protein levels of AQP1 and AQP5 are decreased in inflammatory states [38,39]. Consistent with these, we observed that the protein levels of AQP1 and AQP5 were lower in the lung tissues of allergic mice than in normal control. These diminished protein levels may correlate with injury to alveolar epithelial and endothelial cells [40,41]. It is worth noting that TNF-α has been reported to induce a concentration- and time-independent decrease in the expression of AQP1 and AQP5 [42]. Similarly, IL-13 has also been shown to down-regulate the protein level of AQP5, although the underlying mechanism has not been determined [43]. Consequently, we believed that the increased levels of TNF-α and IL-13 contributed to the decrease in the expression of AQP1 and AQP5, while the decreased protein level of AQP1 and AQP5 could further enlarge the lung inflammation and tissue damage.

AQP5, together with AQP1, is the primary route for osmotic water transport between the capillary and the airspace [38,39], and is fundamental to lung water transport and normal lung function [44]. AQP1 is critically related to lung edema and involved in many inflammatory diseases [45–47]. AQP5 has been proved to be crucial for airway mucus secretion [48]. A decreased protein level of AQP5 has been related to mucus hypersecretion and reduced fluid secretion from the airway epithelium, which leads to high mucus viscoelasticity [49–51]. The alteration in mucus components may hinder its interaction with cilia, and hence, slow its clearance from the lungs [50]. We suspect that the increased protein level of AQP1 and AQP5 in the sevoflurane-treated mice may be related to the sevoflurane-mediated inhibition of mucus secretion.

Evidences show that attenuation of ER stress is associated with increased AQPs expression and improvement of organ function [52,53]. It is known that ER stress and the subsequent downstream signaling have been strongly linked to inflammatory diseases. Many treatments have been focused on alleviating ER stress in controlling inflammation. In the present study, we displayed that treatment with sevoflurane increased the down-regulated protein levels of AQP1 and AQP5 in allergic mice airway and decreased ER stress markers BiP and CHOP. We speculated that the anti-inflammatory role of sevoflurane is related to both direct inhibition of the downstream signaling of ER stress and also ER stress-related AQPs expression.

In summary, our findings suggest that sevoflurane modulated the expression and protein level of AOPs (AQP1, AQP5) as well as inhibited ER stress response in OVA-induced allergic airway inflammation of mice. The present study provides further theory basis from laboratory for the application of the usage of sevoflurane in controlling asthma.

## Abbreviations

AQP: aquaporin
BALF: bronchoalveolar lavage fluid
Bip: heavy-chain binding protein
C/EBP: CCAAT/enhancer binding protein
CHOP: C/EBP homologous protein
ER: endoplasmic reticulum
GAPDH: glyceraldehyde-3-phosphate dehydrogenase
GRP78: the 78kDa glucose-regulated protein
HE: Hematoxylin and Eosin
HRP: horseradish peroxidase
IL: interleukin
OVA: ovalbumin
PBS: phosphate-buffered saline
RIPA: Radio Immunoprecipitation Assay
Th2: T helper 2
TNF-α: tumor necrosis factor-α
